# Combining biofeedback and Narrative Exposure Therapy for persistent pain and PTSD in refugees: a pilot study

This article has been retracted.

**DOI:** 10.3402/ejpt.v3i0.17660

**Published:** 2012-06-25

**Authors:** Naser Morina, Thomas Maier, Richard Bryant, Christine Knaevelsrud, Lutz Wittmann, Michael Rufer, Ulrich Schnyder, Julia Müller

**Affiliations:** 1 Department of Psychiatry and Psychotherapy, University Hospital Zurich, Switzerland; 2 Psychiatric Services of the Canton St. Gallen-North, Switzerland; 3 School of Psychology, University of New South Wales, Sydney, Australia; 4 Department of Psychology, Free University Berlin, Germany

**Keywords:** Refugees, persistent pain, PTSD, treatment, biofeedback, Narrative Exposure Therapy

## Abstract

**Objective:**

Many traumatised refugees suffer from both persistent pain and posttraumatic stress disorder (PTSD). To date, no specific guidelines exist for treatment of this group of patients. This paper presents data on a pilot treatment study conducted with 15 traumatised refugees with persistent pain and PTSD.

**Methods:**

Participants received 10 sessions of pain-focused treatment with biofeedback (BF) followed by 10 sessions of Narrative Exposure Therapy (NET). Structured interviews and standardised questionnaires were used to assess symptoms of pain intensity, pain disability, PTSD and quality of life directly before and after treatment and at 3 months follow-up.

**Results:**

Following the combined intervention, participants showed a significant reduction in both pain and PTSD symptoms, as well as improved quality of life. Additionally, biofeedback increased motivation for subsequent trauma-focused therapy, which in turn was related to larger PTSD treatment gains.

**Conclusion:**

This pilot study provides initial evidence that combining BF and NET is safe, acceptable, and feasible in patients with co-morbid persistent pain and PTSD.

There are an estimated 15.4 million refugees worldwide (United Nations High Commissioner for Refugees [UNHCR], 2011). Due to sequential and longstanding interpersonal trauma such as torture, often experienced in the context of war, refugees are at special risk for suffering from a more complex pattern of trauma-spectrum disorders and appear less responsive to treatment, compared to other victims of traumatisation (Robjant & Fazel, 2010). Research indicates that refugee populations typically report high rates of psychopathology (Steel et al., 2009); with PTSD being especially prominent (Schubert & Punamäki, 2011). Furthermore, these mental health problems persist many years after their first occurrence (Schubert & Punamäki, 2011), often compounded by difficulties with emotion tolerance (Momartin, Silove, Manicavasagar, & Steel, 2003; Zarowsky, 2004) and post-migration living difficulties (Steel et al., 2011). A critical feature that frequently complicates the treatment of mental health in refugees is the concurrent problem of persistent pain (Carinci, Mehta, & Christo, 2010). It is a particularly frequent co-morbid condition of PTSD (Johnson & Thompson, 2008). This specific co-morbidity is especially common in traumatised refugees, asylum seekers and torture survivors (Hinton & Lewis-Fernández, 2011; Silove, Steel, McGorry, & Mohan, 1998). Co-morbidity of both disorders generally results in more severe functional disturbance and reduced quality of life, and has been reported in up to 76% of treatment-seeking traumatised refugees (Dahl, Dahl, Sandvik, & Hauff, 2006; De Jong et al., 2001).

Current models postulate that PTSD and pain are mutually maintaining, because PTSD symptoms can heighten arousal, which leads to increased muscle tension and muscular pain, which can subsequently function as reminders of traumatic experiences, which in turn elicit further PTSD re-experiencing reactions (Carty, O'Donnell, Evans, Kazantzis, & Creamer, 2011; Liedl et al., 2010; Sharp & Harvey, 2001). Despite the observed interplay between pain and PTSD, no studies have been published on treating these co-morbid conditions in this population. Accordingly, there is a need for proof-of-concept studies to determine appropriate treatments to manage the co-morbidity of persistent pain and PTSD.

One proven means of alleviating pain-related distress is a biofeedback-based cognitive behavioural intervention (BF; Morley, Eccleston, & Williams, 1999). BF is a treatment technique by which people learn how to change psychophysiological parameters to improve their health by using signals from their own bodies. Some limited evidence exists demonstrating beneficial effects of BF on posttraumatic pain (Müller et al., 2009; Tatrow, Blanchard, & Silverman, 2003), but the effects are less pronounced than for mono-morbid persistent pain patients. Additionally, it appears to be insufficient as a stand-alone treatment for PTSD (Foa, Keane, Friedman, & Cohen, 2008). A pilot study with traumatised refugees suffering from co-morbid pain and PTSD revealed BF to be well-accepted and exert strong effects on patients’ coping with pain (Müller et al., 2009).

Amongst different PTSD psychotherapies for refugees (Heide, Mooren, Kleijn, Jongh, & Kleber, 2011; Nickerson, Bryant, Silove, & Steel, 2011), Narrative Exposure Therapy (NET; Schauer, Neuner, & Elbert, 2005) is a well-established therapy with strong treatment effects for the reduction of PTSD symptom severity (Neuner, Schauer, Klaschik, Karunakara, & Elbert, 2004; Nickerson et al., 2011; Robjant & Fazel, 2010). NET is a short-term trauma-focused therapy that focuses on imaginary exposure to memories of the traumatic event and the reorganisation of these memories into a coherent chronological narrative. So far, only one study has demonstrated any efficacy of NET in refugees and/or asylum seekers in a Western setting (Neuner et al., 2010).

Taking into account that many refugees suffer from co-morbid PTSD and persistent pain, combining biofeedback for pain with NET may provide additive effects relative to either intervention alone. The use of biofeedback is further indicated for refugees, because many refugees come from cultures in which distress is expressed somatically (Hinton, Pich, Chhean, Safren, & Pollack, 2006) and somatically-based interventions may carry a certain level of face validity. Generally, the first step in evaluating a treatment is to determine its feasibility, acceptance, and safety within a proof-of-concept study, prior to more rigorous testing through controlled trials. To this end, we evaluated the preliminary effects of a combined, pain-focused, 10-session BF program followed by 10-session trauma-focused NET protocol for traumatised refugees. This was an uncontrolled pilot study to examine the feasibility, acceptance, and safety of the combined intervention.

## Methods

### Participants

The study was conducted between March 2008 and October 2009, with approval from the Ethics Commission of the Canton of Zurich. Of all the patients who had been referred to the Outpatient Unit for Victims of Torture and War in the Department of Psychiatry and Psychotherapy (University Hospital of Zurich) over this time, 18 individuals were preselected based on their referral letter indicating co-morbid persistent pain and PTSD, and asked if they would be willing to participate in the study. All these 18 patients committed to the study and fulfilled inclusion criteria, according to our psychiatric and neuropathic examination. The inclusion criteria were: experience of torture/war; current DSM-IV diagnoses of persistent pain (excluding neuropathic pain) and PTSD; and either no psychoactive medication or a stable dose (i.e., participants on medication were required to maintain their dosage for the duration of the trial). Exclusion criteria were: additional pain-/trauma-focused psychotherapy over the course of the study; current psychotic or substance-related disorders; a history of any organic mental disorder; prominent current homicidal or suicidal ideations; severe dissociative symptoms; and any perceived risk of deportation within the next 12 months.

Fifteen participants completed the treatment program.. The majority of the participants were male (60%, *n*=9). Eight participants originated from Turkey (of which six were of Kurdish descent), three from Bosnia, and one each from Sri Lanka (Singhalese), Iraq, Syria and Vietnam. Participants had an average age of 43.1 years (*SD*=6.9) and an average of 9.7 years of schooling (*SD*=4.1), and had lived in Switzerland for an average of 11.0 years (*SD*=5.8). No patient who was asked to participate had to be excluded due to insecure visa status.

Assessments were conducted at four time points: T1 = pre-BF, T2 = post-BF/pre-NET, T3 = post-NET, and T4 = 3 months of follow-up. The assessment and treatment protocols were translated by professional interpreters. Patients completed 10 sessions of manualised BF, as described elsewhere (Liedl et al., 2011; Müller et al., 2009) followed by 10 sessions of Narrative Exposure Therapy (Schauer et al., 2005).

In accordance with the study protocol, psychological assessment and treatment were provided by four postgraduate clinical psychologists who had received special training in the assessment as well as in the application of the manual. All of them participated in weekly supervision sessions dealing with questions regarding assessment and treatment. Neurological assessments were performed by psychiatrists (at least resident level).

### Instruments

The M.I.N.I. Plus version (Ackenheil, Stotz-Ingenlath, Dietz-Bauer, & Vossen, 1999) is a standardised interview that assesses major Axis I psychiatric disorders including somatoform pain disorders according to DSM-IV; this only was used to determine if individuals satisfied inclusion/exclusion criteria. Pain intensity was measured using the self-reported Verbal Rating Scale (item 7 of the SF-36; Ware & Sherbourne, 1992), which assesses current pain levels on a six-point rating scale (*1 = no current pain* to 6 = *extreme current pain*). The self-reported Pain Disability Index (Tait, Chibnall, & Krause, 1990) assesses the impact of pain on a person's ability to participate in essential life activities (ranging from 0 = *no disability* to 10 = *worst disability*). Only those four of seven items relevant to refugees (family/home responsibilities, sexual behaviour, self-care, and life-support activities) were administered. PTSD symptoms were assessed using the Clinician-Administered PTSD Scale (CAPS; Blake et al., 1990). The CAPS is a structured clinical interview that assesses the 17 DSM-IV PTSD criteria. Quality of life was assessed with the WHO self-reported EUROHIS-QOL which has been widely used and validated internationally in many different cultures and languages (Nossikov & Gudex, 2003); it is comprised of eight items that index personal satisfaction with various life domains on five-point rating scales. Motivation for trauma-focused therapy was assessed via six items administered at T1 and T2 that employed a 100 mm Visual Analogue Scale ranging from 0 = *not at all* to 100 = *completely*; (“How big is your motivation for psychotherapy, which focuses on the processing of the trauma you have experienced?”). Cronbach's alpha (*α*=.69) was acceptable.

#### Data analysis

Data were analysed using SPSS 19.0 and were performed on completers only. Time courses were performed using the GLM for repeated measures and paired *t*-tests. Because of the small sample size, missing data were imputed (data missing at each time point: T1 = 1.6%; T2 = 6.7%; T3 = 13.3%; T4 = 26.6%) to maximise the use of information. As data were missing at random (Tsikriktsis, 2005), five complete data sets were imputed applying an EM algorithm (PRELIS) and an average of the imputations was constructed. To determine changes in treatment effects, Cohen's *d* effect size was calculated (Cohen, 1988). Regarding motivation for trauma-focused therapy, subgroups were created to represent highly (*n*=7) and poorly (*n*=8) motivated patients using a median split.

## Results

Generally, the procedure was accepted very well; no patient demonstrated any deterioration. Of 18 patients included in the study, 15 completed all treatment sessions, while two had to be excluded due to life crises unrelated to the treatment protocol (death of a best friend and severe maternal illness) and one dropped out after the third session of BF treatment.

After completion of the BF intervention, there were no significant reductions in pain intensity (*d*=0.45; *t*(14) = 1.47, *p*=.164) or PTSD symptoms (*d*=0.1; *t*(14) = 1.89, *p*=.79). Motivation for trauma-focused therapy increased significantly from pre to post BF with Cohen's *d*=–1.01 and *t*(14) = –3.50, *p*=.004; T1: *M*=5.10, *SD*=2.37; T2: *M*=7.44, *SD*=2.24.

As expected, effect sizes indicated that additional NET had a strong effect on posttraumatic stress symptoms, and moderate effects on pain intensity. Table 1 presents the mean scores at each assessment time for each dependent variable, as well as effect sizes for pre-post-BF, pre-post-NET, post-NET, and 3-month follow-up, and GLM time courses T1–T4 for repeated measures.

**Table 1:** Means, standard deviations, treatment effect sizes and time course (*N*=15 for all time points)

	Means (standard deviations)				Effect sizes (Cohen's *d*)			Symptom time course
			
Variables	T1^a^	T2^b^	T3^c^	T4^d^	T1–T2	T2–T3	T3–T4	Time contrasts (F) GLM

VRS	4.80 (.94)	4.40 (.83)	3.87 (.92)	3.35 (1.12)	0.45	0.61	0.44	12.82*** (3, 42)
PDI	23.40 (9.46)	22.33 (8.31)	20.82 (10.69)	15.39 (9.50)	0.11	0.15	0.53	4.39** (3, 42)
CAPS	83.19 (22.51)	78.47 (22.76)	47.33 (23.87)	48.95 (26.70)	0.1	1.43	−0.01	22.01*** (1.3, 18.39)
QoL	17.88 (4.08)	18.62 (5.79)	19.51 (5.34)	21.47 (6.20)	−0.15	−0.15	−0.37	5.54** (3, 42)

Note: VRS, Verbal Rating Scale (range 1–6); PDI, Pain Disability Index (range 0–40); CAPS, Clinician-Administered PTSD Scale (0–136); QoL, Eurohis Quality of Life (8–40).

a T1 = pre-biofeedback (BF)

b T2 = post-BF/pre-NET

c T3 = post-NET

d T4 = 3 months follow-up.

** *p*<.01

*** *p*<.001.

Figure 1 illustrates the time courses of the outcome variables. As anticipated, a steady reduction in pain intensity and pain disability and an increase in quality of life were observed over time. At follow-up, medium effects were found relative to post-treatment for pain intensity, pain disability, and quality of life, but not for PTSD.

**Fig. 1:** Changes over time of observed variables at four time points (time course). Note: VRS, Verbal Rating Scale; PDI, Pain Disability Index; CAPS, Clinician-Administered PTSD Scale; QoL, Eurohis Quality of Life. Brackets indicating standard deviations.

In order to examine the impact of BF on NET, participants were divided into groups representing high and poor gains in motivation for trauma-focused therapy during BF, using a median split. Patients with strong BF-related gains in motivation exhibited larger decreases in PTSD symptoms during NET than subjects without pronounced gains in motivation (*t*(13) = 3.17, *p*=.007).

## Discussion

The aim of this pilot study was to assess the potential feasibility, acceptance, and safety of combined BF and NET for co-morbid persistent pain and PTSD in refugee trauma survivors.

Regarding the following findings, the combined intervention seemed to be feasible, well accepted, tolerated and safe. None of the patients declined to participate; there were only three drop-outs, none of them related to the intervention; and no patient experienced any exacerbations in pain or PTSD symptoms or any form of personal crisis during the intervention or follow-up period. All outcomes improved significantly after the combined intervention. Improvements in posttraumatic stress symptoms persisted at 3 months of follow-up, and improvements were even more marked for all other measures. Finally, we noted increased motivation for trauma-focused therapy after BF.

In terms of pain response, there was a moderate pre to post decrease in pain intensity. Following NET, there was a moderate reduction in pain intensity, a small reduction in pain disability, and slightly improved quality of life. Conversely, by 3 months of follow-up, there were marked improvements in terms of pain and quality of life. Interestingly, there was no reduction in pain intensity following BF; however, there was noted pain reduction after NET and at follow-up. This pattern concurs with models that PTSD symptoms themselves cause pain to persist, and that reducing PTSD intensity through NET yields a subsequent decrease in pain (Liedl et al., 2010; Sharp & Harvey, 2001). Alternatively, it is possible that the effects of BF were not immediately apparent, and that they only were observed following the additive NET intervention. Given that somatisation is quite frequent among refugees (Aragona et al., 2011; Schweitzer, Melville, Steel, & Lacherez, 2006), a physiologically-oriented approach such as BF may provide refugees with an intervention of strong face validity, because it concurs with their somatic experience of distress, and addresses the significant pain that they experience.

In terms of reducing PTSD, there were marked reductions following NET and these were maintained at follow-up (effect size of 1.45), which is in accordance with previous studies on NET for refugees (Ertl, Pfeiffer, Schauer, Elbert, & Neuner, 2011; Neuner et al., 2004). The question arises concerning the role of BF in preparing refugees for NET. BF may have enabled patients to benefit from exposure treatment, because enhanced pain management may prevent exacerbation of pain during exposure (Wald, Taylor, & Fedoroff, 2004). Furthermore, BF may play a role in establishing the therapeutic relationship that provides stabilisation for refugees, who frequently experience distrust as a result of interpersonal traumatic experiences (Nickerson et al., 2011). It is possible that BF also contributes a sense of mastery or self-efficacy to refugees, which results in greater distress tolerance and an enhanced capacity to manage traumatic memories. In this sense, this finding also might be understood in the context of recent evidence that treating complex PTSD can be optimised by training patients in skills that enhance emotion regulation prior to commencing exposure therapy (Cloitre et al., 2010).

To determine the relative contributions of BF and NET to reductions in pain and PTSD in refugees, it will be essential to conduct randomised controlled trials that allocate refugees to (a) BF, (b) NET, or (c) combined BF and NET. The pattern of findings in this pilot study may be interpreted in terms of the key role of NET; one could conclude that BF was unnecessary because symptom reduction was not observed after this intervention. Additionally, it will be necessary to examine if BF is more efficacious than other forms of preparatory skills training that have been found to be very effective in other trauma populations prior to NET, such as the emotion regulation training incorporated within Cloitre's STAIR program (Cloitre et al., 2010).

One limitation of the current study is that it was an uncontrolled study with a very small sample. Furthermore, we used the CAPS without blinding the assessors; we therefore do not know if their ratings may have been influenced by their assumptions on the efficacy of either intervention. Additionally, as no clear classification or treatment guidelines exist for DESNOS to date, we decided to diagnose persistent pain and PTSD as two distinct co-morbid concepts in our study. However, we are aware that these two disorders are highly interrelated and might be better captured in a single diagnosis, as was suggested for DESNOS (American Psychiatric Association, 1994).

Despite these limitations, the present study provides initial evidence that combining BF and NET is safe, acceptable, and feasible in patients with co-morbid persistent pain and PTSD. Furthermore, biofeedback increased motivation for subsequent trauma-focused therapy, which in turn was related to larger PTSD treatment gains. Given the prevalence of refugees with these co-morbid conditions and the documented impairment these conditions cause (Dahl et al., 2006; De Jong et al., 2001), this first step offers one avenue for controlled trials to test the relative efficacies of these treatment strategies.

## References

[CIT0001] Ackenheil M, Stotz-Ingenlath G, Dietz-Bauer R, Vossen A (1999). *Mini international neuropsychiatric interview* (German Version 5.0.0, DSM-IV).

[CIT0002] American Psychiatric Association (1994). *Diagnostic and statistical manual of mental disorders* (DSM-IV).

[CIT0003] Aragona M, Pucci D, Carrer S, Catino E, Tomaselli A, Colosimo F (2011). The role of post-migration living difficulties on somatization among first-generation immigrants visited in a primary care service. Annali dell'Istituto Superiore di Sanita.

[CIT0004] Blake D. D, Weathers F. W, Nagy L, Kaloupek D. G, Klauminzer G, Charney D. S (1990). A clinician rating scale for assessing current and lifetime PTSD: The CAPS-1. Behavior Therapist.

[CIT0005] Carinci A, Mehta P, Christo P (2010). Chronic pain in torture victims. Current Pain and Headache Reports.

[CIT0006] Carty J, O'Donnell M, Evans L, Kazantzis N, Creamer M (2011). Predicting posttraumatic stress disorder symptoms and pain intensity following severe injury: The role of catastrophizing. European Journal of Psychotraumatology.

[CIT0007] Cloitre M, Stovall-McClough K. C, Nooner K, Zorbas P, Cherry S, Jackson C. L (2010). Treatment for PTSD related to childhood abuse: A randomized controlled trial. American Journal of Psychiatry.

[CIT0008] Cohen J (1988). Statistical power analysis for the behavioral sciences.

[CIT0009] Dahl S, Dahl C. I, Sandvik L, Hauff E (2006). Chronic pain in traumatized refugees. Tidsskrift for den Norske Lægeforening.

[CIT0010] De Jong J. T. V. M, Komproe I. H, Van Ommeren M, El Masri M, Araya M, Khaled N (2001). Lifetime events and posttraumatic stress disorder in 4 postconflict settings. JAMA: The Journal of the American Medical Association.

[CIT0011] Ertl V, Pfeiffer A, Schauer E, Elbert T, Neuner F (2011). Community-implemented trauma therapy for former child soldiers in Northern Uganda: A randomized controlled trial. JAMA: The Journal of the American Medical Association.

[CIT0012] Foa E. B, Keane T. M, Friedman M. J, Cohen J (2008). Effective treatments for PTSD: Practice guidelines from the International Society for Traumatic Stress Studies.

[CIT0013] Heide F. J. J. T, Mooren T. M, Kleijn W, Jongh A. d, Kleber R. J (2011). EMDR versus stabilisation in traumatised asylum seekers and refugees: Results of a pilot study. European Journal of Psychotraumatology.

[CIT0014] Hinton D. E, Lewis-Fernández R (2011). The cross-cultural validity of posttraumatic stress disorder: implications for DSM-5. Depression and Anxiety.

[CIT0015] Hinton D. E, Pich V, Chhean D, Safren S. A, Pollack M. H (2006). Somatic-focused therapy for traumatized refugees: Treating posttraumatic stress disorder and comorbid neck-focused panic attacks among Cambodian refugees. Psychotherapy.

[CIT0016] Johnson H, Thompson A (2008). The development and maintenance of post-traumatic stress disorder (PTSD) in civilian adult survivors of war trauma and torture: A review. Clinical Psychology Review.

[CIT0017] Liedl A, Müller J, Morina N, Karl A, Denke C, Knaevelsrud C (2011). Physical activity within a CBT intervention improves coping with pain in traumatized refugees: Results of a randomized controlled design. Pain Medicine.

[CIT0018] Liedl A, O'Donnell M, Creamer M, Silove D, McFarlane A, Knaevelsrud C (2010). Support for the mutual maintenance of pain and post-traumatic stress disorder symptoms. Psychological Medicine.

[CIT0019] Momartin S, Silove D, Manicavasagar V, Steel Z (2003). Dimensions of trauma associated with posttraumatic stress disorder (PTSD) caseness, severity and functional impairment: A study of Bosnian refugees resettled in Australia. Social Science & Medicine.

[CIT0020] Morley S, Eccleston C, Williams A (1999). Systematic review and meta-analysis of randomized controlled trials of cognitive behaviour therapy and behaviour therapy for chronic pain in adults, excluding headache. Pain.

[CIT0021] Müller J, Karl A, Denke C, Mathier F, Dittmann J, Rohleder N (2009). Biofeedback for pain management in traumatised refugees. Cognitive Behaviour Therapy.

[CIT0022] Neuner F, Kurreck S, Ruf M, Odenwald M, Elbert T, Schauer M (2010). Can asylum-seekers with posttraumatic stress disorder be successfully treated? A randomized controlled pilot study. Cognitive Behaviour Therapy.

[CIT0023] Neuner F, Schauer M, Klaschik C, Karunakara U, Elbert T (2004). A comparison of narrative exposure therapy, supportive counseling, and psychoeducation for treating posttraumatic stress disorder in an african refugee settlement. Journal of Consulting and Clinical Psychology.

[CIT0024] Nickerson A, Bryant R. A, Silove D, Steel Z (2011). A critical review of psychological treatments of posttraumatic stress disorder in refugees. Clinical Psychology Review.

[CIT0025] Nossikov A, Gudex C (2003). EUROHIS: Developing common instruments for health surveys.

[CIT0026] Robjant K, Fazel M (2010). The emerging evidence for Narrative Exposure Therapy: A review. Clinical Psychology Review.

[CIT0027] Schauer M, Neuner F, Elbert T (2005). Narrative Exposure Therapy (NET).

[CIT0028] Schubert C. C, Punamäki R. -L (2011). Mental health among torture survivors: cultural background, refugee status and gender. Nordic Journal of Psychiatry.

[CIT0029] Schweitzer R, Melville F, Steel Z, Lacherez P (2006). Trauma, post-migration living difficulties, and social support as predictors of psychological adjustment in resettled Sudanese refugees. The Australian and New Zealand Journal of Psychiatry.

[CIT0030] Sharp T. J, Harvey A. G (2001). Chronic pain and posttraumatic stress disorder: Mutual maintenance?. Clinical Psychology Review.

[CIT0031] Silove D, Steel Z, McGorry P, Mohan P (1998). Trauma exposure, postmigration stressors, and symptoms of anxiety, depression and post-traumatic stress in Tamil asylum-seekers: Comparison with refugees and immigrants. Acta Psychiatrica Scandinavica.

[CIT0032] Steel Z, Chey T, Silove D, Marnane C, Bryant R. A, Van Ommeren M (2009). Association of torture and other potentially traumatic events with mental health outcomes among populations exposed to mass conflict and displacement. JAMA: The Journal of the American Medical Association.

[CIT0033] Steel Z, Momartin S, Silove D, Coello M, Aroche J, Tay K. W (2011). Two year psychosocial and mental health outcomes for refugees subjected to restrictive or supportive immigration policies. Social Science & Medicine.

[CIT0034] Tait R. C, Chibnall J. T, Krause S (1990). The pain disability index: Psychometric properties. Pain.

[CIT0035] Tatrow K, Blanchard E. B, Silverman D. J (2003). Posttraumatic headache: An exploratory treatment study. Applied Psychophysiolgy & Biofeedback.

[CIT0036] Tsikriktsis N (2005). A review of techniques for treating missing data in OM survey research. Journal of Operations Management.

[CIT0037] United Nations High Commissioner for Refugees (UNHCR) (2011). UNHCR Global Trends 2010. http://www.unhcr.org/4dfa11499.html.

[CIT0038] Wald J, Taylor S, Fedoroff I. C, Taylor S (2004). The challenge of treating PTSD in the context of chronic pain. Advances in the treatment of posttraumatic stress disorder.

[CIT0039] Ware J. E, Sherbourne C. D (1992). The MOS 36-item short-form health survey (SF-36). I. Conceptual framework and item selection. Medical Care.

[CIT0040] Zarowsky C (2004). Writing trauma: Emotion, ethnography, and the politics of suffering among somali returnees in Ethiopia. Culture, Medicine and Psychiatry.

